# Emotion Recognition of Violin Playing Based on Big Data Analysis Technologies

**DOI:** 10.1155/2022/8583924

**Published:** 2022-09-15

**Authors:** Liangjun Zou

**Affiliations:** School of Music, Guangdong Polytechnic Normal University, Guangzhou, Guangdong 510665, China

## Abstract

The rapid development of Internet technology has promoted the vigorous development of the multimedia. As one of the most classic instruments, the violin has been fully developed in its creation, education, and performance. In the face of more and more violin performances, the effective organization and retrieval of these musical works is an urgent problem to be solved, while it is common to classify and organize music based on the emotional properties of the performance. Deep learning is a model based on feature hierarchy and unsupervised feature learning, which has strong learning ability and adaptability. Based on the recurrent neural network (RNN) method, long short-term memory (LSTM) is one of the classic models of deep learning that can effectively learn the characteristics of time series data and achieve effective predictions. Therefore, based on the classical Hevner emotion classification model, this paper proposes an emotion recognition method for dynamic violin performances based on LSTM, which selects acoustic features and classifies the audio acoustic signals contained in the violin performances. In order to verify the effectiveness of this method, this paper carries out data labeled, feature selection, and model test on the actual violin music data by turn. The results show that the proposed method can greatly reduce the training time and improve the prediction accuracy, which reached 83%, higher than the existing methods. Meanwhile, the accuracy and iteration times of violin playing music of different emotional categories are also counted. Moreover, the method is robust to the genre, timbre, and noise changes, and the emotion recognition effect is superior.

## 1. Introduction

With the development of the economy and the improvement of material level of everyone, people begin to constantly pursue the enrichment of the spiritual world, namely, music, art, literature, and music performance. Music is emotional, and music expresses emotions through its sound wave vibrations, lyrics, melodies, rhythms, etc. It also relates to our emotional activities. It is a mental process that arises in the process of human interaction with music, namely, various human emotional factors. The emotion of music has a lot of impact on our lives. On the one hand, we could receive emotional messages and have a better musical experience form listening to music. On the other hand, music can express emotions, stimulate emotional experiences, have an impact on people's hearts, trigger brain physiological activities, and affect people's behavior and decision-making. Violin is one of the most classic instruments, both timbre and performance form are very popular with the public, violin performance in the musical art expression occupies a vital position, and in the contemporary open and free social environment, violin creation, education, and performance have been fully developed.

With the development of Internet music, a large number of songs are released through the network and stored in large digital music databases, and the organization and retrieval of online music works have attracted more and more attention from industry and academia. At the same time, the requirements of people for music are not only fine-sounding and spending time but also fit our emotional needs by seeking resonance from emotional performance of music. Given the consensus that music expresses and evokes emotions, the need to organize and retrieve music based on the emotional properties of music is objectively existent. Studies have found that the most commonly used word to retrieve and describe music is the emotional word. In order to achieve emotion-based music retrieval, it is often necessary to label the emotions of musical works. Using artificial methods to mark the emotion of a large number of music, not only the workload is huge but also the quality cannot be guaranteed, and the work efficiency is low [1, 2]. Therefore, it has become an inevitable choice to study the automatic recognition technology of musical emotion and realize the automatic emotion labeling of musical works [3, 4].

Automatic recognition of musical emotion refers to the process of constructing a computational model based on the audio data of music and other related information to realize the automatic identification of musical emotion [5]. Making music correspond to various emotions and provide services to those who need it is the aim of music emotion recognition [4, 6]. Musical emotion recognition technology involves many fields, namely, musicology, psychology, music acoustics, audio signal processing, natural language processing, and deep learning [7, 8], and it is a multidisciplinary and interdisciplinary research field [9].

Deep learning is one of the more popular artificial intelligence methods in recent years, which has the advantages of strong learning ability, wide coverage, good adaptability, and strong portability [10, 11]. It has attracted in-depth research by many experts and scholars and has been widely used in image recognition, image segmentation, natural language processing, and other scenarios and has achieved great success [12, 13]. At the same time, more and more scholars are also trying to apply deep learning technology to the field of musical emotion recognition [14]. The method of deep learning gets the relationship between the underlying features of audio and higher-level concepts from audio data [15, 16]. The great challenge facing musical emotion recognition is that there is a difference between the characteristics of the audio signal and the emotional semantics of the music that is difficult to describe with physical parameters, and emotion recognition through deep learning may be able to cross this difference [17]. Convolutional neural network (CNN) [18, 19] and RNN have demonstrated their excellent performance in many music classification tasks.

The emotional expression of music is dynamic, the emotions reflected at different moments are different, and the subsequent emotional expression is based on the previous emotional expression, and this feature is less considered in the existing research on musical emotion recognition [20]. LSTM is specially designed to solve the long-term dependence problem of general RNN, which can capture the change patterns in the sequence data and predict the future trend of the data [21]. Therefore, this paper uses the LSTM method to extract features and identify emotions of violin performances and verifies them with actual data. Experimental results show that the accuracy of emotion recognition proposed in this paper is relatively high compared with other methods, which has superiority [22, 23].

This paper uses deep learning technology to identify the dynamic emotions of the violin performance, which makes up for the fact that the dynamics of the emotions in the violin performance are not considered in the existing research and have superior performance. This paper is divided into five chapters. The first section explains the necessity and significance of applying deep learning to the emotional recognition of violin performance. The second section introduces and summarizes the current literature and research status of musical emotion recognition. In the third section, we describe the overall process and scheme of violin performance emotion recognition using LSTM method from three aspects: musical emotion representation model, musical emotion characteristic recognition, and violin performance emotion recognition based on LSTM. In the fourth section, the method proposed in this article is verified by using actual data, and the corresponding results are discussed and explained. The fifth chapter briefly summarizes the research content of this article, language processing, and other scenarios and has achieved great success.

## 2. Literature Review

The study of musical emotion recognition began in the 1960s and has been around for decades. At the beginning of artificial intelligence, some people proposed the relationship between music content and emotion. Later, universities and research institutes have carried out relevant research. In recent years, with the development of artificial intelligence, the research on musical emotion recognition has made rapid progress and has been successfully applied in various fields, namely, music emotion retrieval, artistic performance of music emotion recognition, and intelligent space design. The recognition of musical emotion is a pattern recognition, and its recognition process requires the data to be correctly mapped from the high-dimensional musical feature space to the low-dimensional emotional space.

According to the differences in the main objects of research, the existing musical emotion classification can be divided into the following three categories: one is the emotional classification of the audio signal based on the melody of the music itself, one is the emotional classification of text information such as lyrics and comments based on the music, and the other is the emotional classification of multimodal fusion based on the two modes of audio and text. According to different research methods, music emotion classification methods can be divided into the following three categories: the first is emotion classification based on existing or self-expanded emotion dictionaries; the second is emotion classification based on machine learning methods; the last is emotion classification using deep learning methods. Next, this section reviews and summarizes the existing literature research.

Hu, Choi, and Downie proposed a multimodal music emotion evaluation model [24], which not only considered the original sound of music but also analyzed the impact of multimodal classification methods on the number of training samples and the length of audio clips. At the same time, it also added music lyrics and online user comments on music as reference standards. An, Sun, and Wang obtained the lyrics of popular music as the text features of music and used the Bayesian classification model in machine learning to classify the emotion of music. The results showed that the accuracy of music emotion classification was ideal, which proved the effectiveness of this method in the process of signal research [25]. Du, Lin, and Sun collected the spectrum and carried out image learning and training, so as to improve the accuracy of the classification model [26]. Jakubik and Halina used the gated recurrent unit (GRU) model to learn the features of audio and then used the support vector machine (SVM) to realize music emotion classification. The experimental results proved that this feature learning method has better classification performance than the high-level audio features based on expert domain knowledge [27]. Gupta, Dileep, and Thenkaniditoor used the traditional machine learning method SVM to classify music [28].

In addition, some scholars found that the combination of neural network model and feature sequence can strengthen the correlation of time series in the process of data classification and obtain better classification results. Therefore, Huang, Chou, and Yang realized the highlighting of emotional focus features and applied them to CNN and attention mechanism [29]; Mirsamadi, Barsoum, and Zhang used the short-term signal characteristics related to emotion in audio to distinguish the emotion of the interlocutor, which was applied to the convolutional neural network and AM (attention mechanism) [30]; Zhang, Xu, and Cao combined samples with CNN to enhance the classification accuracy of the model from the perspective of sample research [31]. Liu, Chen, and Wu used CNN for music emotion recognition and achieved good classification results on two public data sets [32]. Tzirakis et al. proposed a new end-to-end method to recognize the emotional polarity of songs from audio and lyrics through deep neural network, with an accuracy of 80%, but this method only divides musical emotions into positive and negative emotions [33]. Li, Xian, and Tian fused the deep bidirectional LSTM model with the extreme learning machine [34] and predicted the real-time emotional state of music clips. Dong et al. proposed a bidirectional convolution recursive sparse network, whose input is the spectrum of music [35]. The existing research does not consider the dynamics of music. There are few studies on music emotion recognition for a certain category of musical instruments. At present, the research on music emotion recognition is mainly based on audio, lyrics, and related tag data on social media. Compared with music with lyrics information, its emotion recognition lacks the assistance of text information. At the same time, the emotional characteristics of playing music are often dynamic, so this paper proposes an emotional recognition model of violin playing music based on LSTM to make up for the gap of existing research.

## 3. Emotion Recognition of Violin Playing Based on LSTM

### 3.1. Music Emotion Expression Model

Emotion is a psychological process of multi-component, multi-dimensional, and multi-level integration. Moreover, emotion is the essential feature of music. The mathematical model of music emotion bases on the psychological model research. Combined with the research of music theory, music psychology, and art emotion, the performance, transmission, and cognitive behavior process of music emotional information have the following typical characteristics:

The first characteristic is subjectivity. Music performances are the reflection of reality through the tortuous mapping and selection of the artist's mind. It has a high degree of subjectivity. Due to the differences in culture, environment, habits, and personality, the psychological structure at both ends of emotional information transmission is often in different modes. This subjectivity reflects all links of the emotional transformation system.

The second characteristic is hierarchy. In people's cognition of the characteristics of music, style and emotion are the highest and deepest cognition. After this stage, music will be internalized into a psychological feeling of people, affect people's mental state, and may become an inspiration element for composers to recreate music.

The third characteristic is objectivity. Pure emotion only exists in people's hearts. To make others feel the same, we must use the artistic symbols with the common structure of emotion to express it.

The fourth characteristic is fuzziness. Emotion is the implicit knowledge of art form, which can be deconstructed by multi-source information fusion method based on expressive symbol system, and these artistic symbols are basic material materials that can be measured, simply perceived, or inferred.

The fifth characteristic is integrity. In music creation and appreciation, it is not to express and grasp emotions from independent notes but to express and experience the role of each note in the theme emotion on the whole.

The last characteristic is sportiness. Human emotions are moving, and each emotion has a process of production, development, and calming down, and this kind of movement characteristics will also exist in the time axis of artworks.

Based on the above summary of music emotion characteristics, researchers have given a variety of music emotion classification models from different research perspectives. At present, the classification of emotional categories mainly includes discrete representation and continuous dimension representation. Among them, discrete emotion describes emotion as discontinuous and discrete emotion category labels. According to the common degree of emotion, discrete emotion can be divided into basic category and extended category. Some researchers also call it primitive emotion and derived emotion. Just as the three primary colors can be mixed to produce other different colors, derived emotion is mixed from the changes of basic emotion. At present, Hevner's emotional model is widely recognized at home and abroad. By analyzing and studying artistic forms such as music, he accurately defines the attributes of emotion and uses the ring structure to express emotion and then divides the ring into eight sectors with typical representative meanings. Each category has a representative adjective: dignified, sad, dreamy, serene, graceful, happy, exciting, and vigorous. In this circular structure, there is a progressive relationship between each two adjacent emotions, so the emotional change can smoothly transition in the adjacent emotions before or after it, as shown in Figure 1. Discrete emotion expression is simple and clear, which is convenient for computer recognition in our research work, but emotion is human subjective feeling after all, and it is difficult to accurately express everyone's emotional state in practical application with certain and classified emotions.

Continuous emotion believes that there is a changeable measure of emotion in a certain nature, so emotion is described as a point in a multidimensional emotional space, each dimension corresponds to a psychological representation of emotional space, and each dimension is described by continuous real numbers. Therefore, continuous emotion is also more applied to standard prediction or fitting problems. At present, the commonly used continuous emotion model is the valence arousal emotion model proposed by Russell. In the V-A model, emotional state is a point distributed in a two-dimensional space containing valence and arousal, while the vertical axis represents arousal and the horizontal axis represents valence. In general, the valence reflects the positive and negative degree of emotion. The higher the value is, the higher the positive degree of emotion is; on the contrary, the negative degree is higher. The degree of arousal reflects the intensity of emotion. The greater the arousal value, the higher the intensity of emotion, and vice versa. The V-A emotion model is shown in Figure 2.

### 3.2. Music Emotion Feature Recognition

The purpose of recognizing music emotion is to enable computers to recognize music emotion automatically through multidisciplinary and multidisciplinary cooperation, which equips the computers with the ability of music emotion recognition. Through computer analysis and processing of music features, the physical acoustic space of music segments is corresponding to people's emotional space to realize emotional recognition.

Generally speaking, the emotion of music can be obtained through the analysis of lyrics, social labels, and audio signals. Although violin playing music does not contain lyrics and other information, its most significant feature is the audio acoustic signal. The rhythm, melody, and loudness of different playing music can carry different musical emotional information. People cannot analyze the characteristics of its lyrics, do not pay attention to the emotional label of the performance, but they can obtain the emotional information of the music only through their own feelings of the melody. Therefore, music emotion recognition based on audio signal is also regarded as the best method to recognize the emotion of violin playing music. It is based on a large number of statistical learning of music emotion and classifies the recognized music features through some emotion classification methods and finally recognizes the music emotion.

Music emotion recognition based on audio signal can be completed through acoustic feature selection, audio segmentation, audio recognition, audio classification, and other steps. On the whole, the audio content of music can be divided into three levels: the lowest physical sample set, the middle acoustic feature set, and the highest semantic set. In the physical sample set, music audio exists in the form of media stream. In the middle layer, we can automatically extract acoustic features from audio data, namely, physical features (such as fundamental frequency and amplitude) and user perceptible features (such as tone and loudness). At the highest level, it is the semantic information of music, that is, the conceptual description of music audio content.

Therefore, after extracting the acoustic features of music by establishing a mathematical model of the non-stationary complex signal of audio signal and using the corresponding classification and prediction model to establish the mapping relationship between acoustic features and music emotion space, the emotion recognition of violin playing music is realized.

### 3.3. Emotion Recognition of Violin Playing Based on LSTM

Deep learning is a method based on feature hierarchy and unsupervised feature learning. It has all the excellent feature learning ability because of many hidden layer, and the learned features have a more essential description of the data. Compared with the traditional machine learning model, the music emotion recognition model based on deep learning has two advantages. First, the performance of the deep learning model will increase with the increase of the amount of training data. Secondly, the model based on deep learning can automatically extract appropriate features from the data. Deep learning is based on neural networks. RNN has memory, parameter sharing, and turing completeness, so it has certain advantages in learning the nonlinear characteristics of sequences. However, with the deepening of the network layer, RNN only obtains the information of the previous node; it cannot store the output of the network far away from the current time, which will cause the gradient to disappear. In order to solve gradient disappearance and gradient explosion, experts and scholars proposed LSTM network, which was widely used in time series prediction for a period of time.

Violin performances and emotional labels do not have a one-to-one correspondence in time domain, and the expression of emotion in violin performances at a certain time is the accumulation of previous music content. Most previous models are one-to-one mapping from acoustic features to emotional labels. Violin playing are actually temporal data, and the effect of emotional classification is superimposed. In other words, their subsequent feelings are based on the emotional foreshadowing in front. So LSTM is an appropriate method to deal with the above problems. Therefore, this paper uses Hevner emotion model to express the dynamic emotion in music and proposes a dynamic violin performance emotion recognition method based on LSTM.

LSTM is an improvement of RNN model to solve the effect of gradient disappearance. This improvement is mainly manifested in adding long-term and short-term memory units to the RNN hidden layer, adding gating structure, introducing sigmoid activation function, and combining with the original tanh activation function of RNN. LSTM solves the problems of short-term dependence and long-distance dependence. The three gating units of LSTM are input layer, hidden layer, and output layer, which together constitute the input part of the model.

1. Input layer. It is a full connection layer. The network first pre-processes the data to meet the input data format requirements. The value *i*_*t*_ of the input gate and the candidate state value $\overset{\sim }{C_{t}}$ of the input cell can be calculated as follows:

(1) $$\begin{array}{c} i_{t}=\delta \left(W_{i}^{*}\left(X_{t},h_{t-1}\right)+b_{i}\right), \end{array}$$

(2) $$\begin{array}{c} {\tilde{C}}_{t}=\tanh\left(W_{c}*\left(X_{t},h_{t-1}\right)+b_{c}\right). \end{array}$$

While **W** and **U** represent the weight matrix during calculation; *b* represents the offset vector; *σ* indicates activation function *sigmoid*.

(2) Hidden layers. It is a recurrent neural network containing multiple LSTM neurons. In this network structure, the activation function selects *σ* and tanh_;_ at time *t*, the *sigmoid* of the forgetting gate and the cell of the mathematical expression of the updated value can be written as:

(3) $$\begin{array}{c} f_{t}=\delta \left({W_{f}}^{*}\left(X_{t},h_{t-l}\right)+b_{f}\right), \end{array}$$

(4) $$\begin{array}{c} C_{t}=i_{t}^{*}{\tilde{C}}_{t}+f_{t}^{*}C_{t-1}. \end{array}$$

(3) Output layer. The final output of the model is obtained by mapping multiple output results of the hidden layer to the full connection layer. In the network structure of this layer, the final output results calculated are as follows:

(5) $$\begin{array}{c} O_{t}=\delta \left(W_{O}*\left(X_{t},h_{t-1}\right)+b_{o}\right), \end{array}$$

(6) $$\begin{array}{c} h_{t}=O_{t}*\tanh\left(C_{t}\right). \end{array}$$

Based on the LSTM method, in Figure 3, this paper constructs the basic framework of emotion recognition of violin playing music. First, the training set is constructed, and the emotion of violin playing music is labeled. Then, the characteristics of the music are extracted and selected. Finally, the LSTM method is used to recognize the emotion in the feature space of the music to get the final emotion label. LSTM method plays a great role, which not only realizes the mapping from music to features but also realizes the mapping from music to emotion model. It is the core part of the whole research framework.

## 4. Result Analysis and Discussion

In order to verify the effectiveness of the method, this paper selects 500 violin performances for experiments. These violin playing are downloaded from the Internet music library, and their data formats are adjusted to the format required by the experiment. At the same time, the characteristics of music are sorted out from the perspective of music theory. Hevner model is an internationally recognized music emotion classification model, which divides music emotion into eight categories. So Hevner model is selected in the experiment. Firstly, we describe the emotions of these violin performances according to the Hevner emotion classification model. We selected 300 violin performances as the training set for LSTM model. The distribution of different categories of violin performances is shown in Figure 4. The horizontal axis represents eight categories in Hevner emotion classification model.

The first step is to divide the existing violin playing music files into multiple segments.

The second step is to extract the features of each music and transform them into the feature vector of the music.

The third step is to input the extracted feature vector into the classification cognitive model and train the LSTM model.

In this experiment, the input of the model is the music feature extracted from the violin playing music, and the output of the model is the emotion category predicted according to the music feature.

The efficiency of violin music emotion recognition based on LSTM model can be evaluated by accuracy, precision, recall, and F1 score. These indicators are classic evaluation indicators in the field of machine learning and deep learning. The calculation principle of these indicators is mainly based on the confusion matrix, as shown in Table 1. Where FP and TP represent the number of samples of false positive class and true positive class, respectively, FN and TN represent the number of samples of false negative class and true negative class, respectively.

The accuracy rate represents the proportion of the number of correct recognition in the total sample, and its formula is as follows:

(7) $$\begin{array}{c} ACC=\frac{TP+TN}{TP+TN+FN+FP}. \end{array}$$

The precision rate represents the proportion of identified positive classes correctly in all identified positive classes, and its formula is as follows:

(8) $$\begin{array}{c} PRE=\frac{TP}{TP+FP}. \end{array}$$

Recall rate refers to the proportion of those correctly identified as positive in all actual positive, and its formula is as follows:

(9) $$\begin{array}{c} REC=\frac{TP}{TP+FN}. \end{array}$$

F1 score takes into account the precision and recall of the model in the calculation process, and its formula is as follows:

(10) $$\begin{array}{c} F1=\frac{2*REC*PRE}{REC+PRE}. \end{array}$$

In the above experiment, from the Figure 5, we could see that the recognition accuracy of the LSTM model reaches 83% when it is trained to 50th steps, and the network converges.

Next, we use the trained model to recognize the emotion of 200 violin music in the test set. In general, the longer the music, the more emotional information it carries, and the greater the emotional fluctuation of music. Therefore, for longer music, the accuracy of emotional recognition will decline. Therefore, this paper compares the accuracy of emotion recognition of different lengths of music. The results are shown in Figure 6.

Violin music of different emotional categories has different feature expressions, so there will be differences in the process of emotional recognition. Therefore, this paper shows the accuracy of emotional recognition of different categories of music in Figure 7(a). From the figure, we can see that the accuracy of emotional recognition of music with emotional categories of grace is relatively high, while the accuracy of emotional recognition of music with emotional categories of serene and happy is relatively low.

At the same time, we get the number of iterations of different emotional categories as shown in Figure 7(b). It can be seen from the figure that the music of these eight emotional categories can reach stable states and high accuracy after 40–55 iterations.

Some experts and scholars have applied machine learning, CNN, RNN, and other technologies to music emotion recognition in the existing research. In order to further verify the effectiveness of this method in this paper, the above-mentioned methods are used to conduct experiments with the data in this paper, and the evaluation is carried out from the four perspectives of ACC, PRE, REC, and F1 score. The specific evaluation results can be seen in Figure 8. According to the results in Figure 8, the emotion recognition model of violin playing music based on LSTM has great advantages, and its four evaluation indicators are better than other methods. Secondly, CNN and RNN have better effect on emotion recognition, while the effect of SVM based violin music emotion recognition method is relatively general, which further verifies the good adaptability and feasibility of deep learning applied to violin music emotion recognition method.

At the same time, we can see the iteration times of violin playing music trained by different neural network methods from Figure 9. SVM is one of the most classical methods in machine learning. The model training process does not involve the iteration of the network layer, so the data related to SVM is not involved in Figure 9. Compared with CNN and RNN methods, LSTM method has higher recognition accuracy after 55 iterations, and the accuracy in the iteration process is better than the other two methods. The accuracy of CNN and RNN is close, and its accuracy continues to improve with the increase of iteration times. The effectiveness of this method is further verified from the timeliness and accuracy.

## 5. Conclusions

At present, higher requirements are put forward for retrieval technology, and people are no longer satisfied with relying on the author and song name to realize song search, but they hope to screen their favorite songs through the emotion conveyed by the music. Artificial intelligence method shows more advantages in emotion recognition. Therefore, we can consider the deep learning technology to realize the emotional recognition of violin playing music. So this paper analyzes the common emotion classification models and selects the appropriate emotion model based on the characteristics of violin music, as well takes into account that violin music and emotion labels do not have a one-to-one correspondence in time domain. This paper uses LSTM method to dynamically analyze the characteristics of time series data in music, so as to realize the emotional recognition of violin playing music. At the same time, this paper selects 500 violin performances and classifies emotions according to the Hevner emotion classification model. Moreover, the method proposed in this paper is used for experimental verification, and the experimental effect is evaluated from the perspective of multiple evaluation criteria such as accuracy, precision, recall, and F1 score. From the experiment, it can be concluded that the method proposed in this paper is superior to the previous music emotion recognition methods, such as machine learning, CNN, and RNN. At the same time, this paper also shows and compares the recognition effect of this method from the perspective of the number of training iterations and the recognition accuracy of different types of music. We can conclude that LSTM method has strong adaptability and feasibility in the emotional recognition of violin playing music. CNN, RNN, and LSTM methods are particularly adaptive and superior. In future research, we will consider combining the characteristics and advantages of these methods to improve the accuracy of violin music emotion recognition.

## Figures and Tables

**Figure 1:** Hevner emotion model.

**Figure 2:** V-A emotion model.

**Figure 3:** Framework of violin performance emotion recognition.

**Figure 4:** Music distribution.

**Figure 5:** Effect evaluation of training model.

**Figure 6:** Accuracy of emotion recognition for violin concertos of different lengths.

**Figure 7:** Accuracy and training times of emotion recognition of different types of music.

**Figure 8:** Effect evaluation of different methods.

**Figure 9:** Training times of different methods.

**Table 1:** Confusion matrix.

Predict|real	True	False
True	TP	FP
False	FN	TN

## Data Availability

The authors declare that the research was conducted in the absence of any commercial or financial relationships that could be construed as a potential conflict of interest.
